This article has been retracted.

# Perception Research of Artificial Intelligence in Environmental Public Health Physiotherapy Nursing for the Elderly

**DOI:** 10.1155/2022/2124710

**Published:** 2022-09-10

**Authors:** Min Shi, Huadong Peng, Yuanxing Lin, Yiming Ma, Yanxin Qi

**Affiliations:** ^1^School of Education, Fuzhou University of International Studies and Trade, 350000, China; ^2^Nanjing Institute of Technology, 210000, China

## Abstract

This perceptual study focuses on developing artificial intelligence for elderly care design. It analyses and discusses the role of artificial intelligence in elderly care and its application to physiotherapy care. Artificial intelligence, as an emerging disruptive technology, is releasing the enormous energy accumulated in the technological and industrial revolutions, profoundly transforming how humans produce, live, and think about the world. Economic development and social progress are significantly impacted by it, and it has a great deal of practicality and broad application scope. Although there is a basic consensus in the 18 public understanding of AI, there is still some ambiguity and misunderstanding, knowing what is happening without understanding why. As a result, it is necessary to systematize and gain a comprehensive understanding of this concept and its associated practices.

## 1. Introduction

There has been significant progress made in the application of artificial intelligence to the field of medical care. However, the vast majority of people do not understand what artificial intelligence (AI) is, what medical care is, what kinds of medical care are necessary for elderly patients, or what effect AI-based physiotherapy care has on patients' mental and physical well-being. In this context, a perceptual study of the design of AI care for the elderly will help establish an appropriate social, moral, and world view, as well as provide a solid foundation for constructing core socialist values [1–3].

The past few years have seen the introduction of intelligent environment public health care robots both in the United States and in other countries. The elderly engage in conversation with the robot, and both the conversation and the data transfer are utilized for remote consultations as well as some straightforward environmental and public health checks. Despite this, the majority of research has concentrated on either broad definitions of AI or the effects of AI on the economy. We are not aware of any artificial intelligence (AI) products that offer specialized services catered to senior citizens. In addition, there is a paucity of published, professional research that points to the social significance of AI physiotherapy care for the elderly. A general definition of “artificial intelligence” would be too simplistic, but an analysis of the characteristics of artificial intelligence combined with perceptual engineering would make it possible to conduct an in-depth study of the topic, reflecting the level of rigor of the study [4, 5].

The topic of artificial intelligence is currently being covered in a significant number of articles across the domestic web. There are a number of well-known papers on the subject of artificial intelligence, such as “Application of Artificial Intelligence in Health Care,” “Consensus, Differences, and Problems in Artificial Intelligence Education: Content Analysis Based on Four Sets of Standard Documents,” and “Research on the use of intelligent caregiving robots in the home – from the perspective of empty nesters' environments” [6–8]. Due to the fact that these discussions and research are primarily conceptual descriptions of how artificial intelligence is applied to caregiving robots or other fields [9, 10], there is no systematic discussion or research on artificial intelligence in the environment pertaining to public healthcare.

Analyses and polls were the primary research approaches utilized for this investigation. The research investigates the beginnings and evolution of artificial intelligence, as well as its definition and concepts. It also compares AI to machine learning and explores the distinctions between the two. In addition to that, the study investigates the various forms that artificial intelligence can take. Second, the study describes the sensory characteristics of the elderly and the potential need for AI physiotherapy care based on the results of the survey in conjunction with perceptual engineering. These findings were derived from both sources. Following that, an examination of the function of AI in physiotherapy for the elderly is presented. In the final section, a sociological analysis is used to investigate the factors that are contributing to the rapid advancement of artificial intelligence in modern society.

## 2. Theoretical Research on Artificial Intelligence

### 2.1. Definition of Artificial Intelligence

The intelligence displayed by machines that have been created by humans is referred to as “artificial intelligence” (AI), which is an abbreviation of the term. Research into artificial intelligence has been conducted in a vast number of fields, including natural language processing, machine perception, machine communication, and creativity, amongst many others. The intelligence that can be exhibited by machines that have been designed and built by humans is referred to as artificial intelligence (AI). Taking a look at Figure 1 makes it abundantly clear that artificial intelligence and machine learning are subcategories of the larger category of artificial intelligence and that deep learning is a subcategory of machine learning [11, 12].

### 2.2. The Development of Artificial Intelligence

Since the advent of the very first computer, advances in artificial intelligence have been steadily being made over the course of the past more than half a century. During this time period, the industry has gone through three distinct periods of expansion. In the study, the development of artificial intelligence over the course of history is dissected, along with an analysis of the factors that led to each technological boom and the challenges that accompanied those booms [13–15].

The first boom, which occurred between the years 1950 and 1960: in the 1950s, computers were used in the process of finding and deducing solutions to a wide variety of problems. This trend continued into the 1960s. As a result of the limited computing power of computers at the time, they were frequently jokingly referred to as artificial intelligence that could only solve problems involving playthings. This was a result of the limited computing power of computers at the time. As a direct consequence of this, during the 1960s they went through a period of withdrawal.

The second boom, which occurred between the years 1980 and 1990: since the 1980s, the knowledge of a large number of subject matter experts has been entered into the computer, which then determines the answers based on the questions that the user has asked. When diagnosing diseases, where an incorrect conclusion could be reached as a result of an incorrect judgment in any one of the successive problems, this system was utilized. An incorrect conclusion could be reached as a result of an incorrect judgment in any one of the successive problems. In addition, the sum total of human knowledge is unfathomably large, and it would be physically impossible to input all of that information into the computer in the appropriate sequence. As a direct consequence of this, the idea ultimately became impossible to implement and fizzled out in the 1990s.

The third boom (from the year 2000 to the present): computers have gotten significantly more powerful as a result of developments in semiconductor technology, which has led to these advancements. In addition, the price of semiconductors has been going down, which has made it more affordable to store data in the cloud. As a direct result of the cloud's capability to collect large amounts of data from locations all over the world, significant strides have been made in the field of artificial intelligence (AI), leading to significant amounts of overall progress. In machine learning, big data is used to teach a computer how to learn the eigenvalues of information, whereas in deep learning, big data is used to teach computers how to understand the eigenvalues of information, which is referred to as “eigen expressions learning.” Both types of learning make use of the same amount of data. Both unsupervised and supervised learning are predicated on the idea that adding more information can result in improved performance.

Over the course of the last few years, developments in semiconductor technology have brought about both an increase in functionality and a decrease in prices. It provides an environment that is ideal for the development of artificial intelligence because it makes storing and processing large amounts of data more accessible. There is no reason for us to be concerned about a slowdown in the growth of artificial intelligence at this time because of the advancements that have been made in the field of information technology. On the other hand, we ought to be concerned that an excessive development of artificial intelligence will be harmful to society. This is because artificial intelligence has the potential to create unintended consequences.

What is the most significant difference between conventional methods of machine learning and the most recent cutting-edge methods of deep learning that are currently accessible? How is it possible for artificial intelligence to differentiate between a pig, a horse, and a cat when it comes to recognizing animals in pictures? In the past, human analysis was used as the foundation for machine learning in order to determine the most distinguishing characteristics of a variety of animals. This was done with the goal of improving animal classification. The position of their ears and eyes, the size of their eyes, and the color of their ears were some of these characteristics. Because of this, the machine was able to acquire the ability to judge in addition to its classification capabilities, which enabled it to develop its own model for classification.

As can be seen in Figure 2, the evolution of artificial intelligence can be broken down into three distinct phases: the first phase began in 1956, when artificial intelligence was first developed; the second phase, which developed expert systems in the 1980s; and the third phase, which developed deep learning in 2006. Deep learning is a neural network-based approach to machine learning that was first presented in 2006. It is credited with kicking off a new era in artificial intelligence as a result of the rise in the availability of big data and computing power (GPUs for matrix operations) [16, 17]. Deep learning was first presented in 2006. Deep learning is credited with kicking off a new era in artificial intelligence as a result of the rise in the availability of big data and computing power.

### 2.3. The Chip of Musk

In theory, Neuralink chips could potentially treat conditions such as paralysis, strokes, and damage to the brain. Musk, the richest person in the world, claims that Neuralink's brain-machine interface will solve the problem of brain and spinal injuries within the next decade. Musk took to Twitter not too long ago to reiterate that his company is having trouble overcoming obstacles, such as finding a treatment for paralysis. In an ideal scenario, neurolinks in the motor cortex and sensory cortex of the brain should be able to restore function throughout the body by connecting neurolinks in the spinal cord with weak or broken connections in the neck and spine [18–20].

The complexity of this electronic, mechanical, and software engineering challenge for Neuralink devices is comparable to that of smartwatches, CNC machines, and surgical robots.

Microchips that can be surgically inserted into human skulls are the focus of Neuralink's research and development efforts. The device is able to read and stimulate the brain thanks to the tiny wires and electrodes that extend outward from it in the direction of the brain. Musk is also of the opinion that Neuralink has the potential to treat a variety of neurological conditions.

The Link V0.9, which comes in the form of an implantable chip, can be placed inside of a piglet. The chip is about the size of a coin and has a diameter of about 8 millimeters. This chip has a long battery life, supports remote data transmission, can sense temperature and pressure, and can collect and transmit neural discharge signals. Other features include the ability to sense temperature and pressure. The implementation of Link V0.9 is the primary focus of the public's concern at this time. The implantation of the Link V0.9 takes significantly less time and does not require the use of anesthesia in comparison to conventional hospital surgery. Additionally, the robot that performs the procedure does all of the work.

## 3. An Analysis of the Perceptual Imagery of the Human Body of the Elderly

As we age, our cornea begins to lose its luster, and its ability to refract light also decreases; the function of our pupil sphincter decreases, causing our pupils to narrow, and this results in a decrease in the amount of light that enters our eyes; the lens becomes cloudy and yellow; and the retina gradually begins to lose its visual receptor cells. All of these changes can be attributed to the natural process of aging. As a consequence of a series of events that resulted in a decrease in physiological regulation, there have been direct repercussions for the manner in which the body processes light and dark, space, color, and information. These alterations have all taken place.

Alterations in the clarity of vision: at age 60, the contrast between the target and the background is equal to two; after that, the decay rate accelerates exponentially, reaching six when the subject is 80 years old. This assumes that the level of visibility was the same at age 20.

There are many different ways that light and dark can be perceived, including once a person reaches the age of 13, their ability to adapt to shifting patterns of light and dark begins a slow and steady decline, with the rate of decline depending on the individual.

Vision problems: as people get older, they frequently have trouble seeing things in front of them because their peripheral vision decreases. This is one of the changes that occur in spatial vision. People of advanced age have a diminished capacity to observe objects in distance and stereo, which renders it impossible for them to determine the height and distance of objects with any degree of precision. If your visual acuity is not as good as it used to be, it is possible that you will not be able to differentiate between the various objects in the same clear manner. This will have an effect on how you perceive the depth of space.

Changes in color vision result from the lens's ability to selectively absorb blue light as it yellows and becomes cloudy with age. Because of this, the ability of older people to distinguish blue from red and green is significantly diminished as a result.

Alterations to one's capacity to process visually presented information: the ability of older people to process visual information, such as visual search and coding, is impaired because they require more time to locate a “9” in a “6” matrix, and the interval between two flashes is long enough to differentiate between them.

The complications and diseases that are associated with age and environment are listed in Table 1.

It is common for the elderly to have reduced visual abilities. Studies have indicated that the elderly prefer a viewing angle of 0.75 degrees at a sight distance of 43 cm, corresponding to a word height of 5.62 mm. This is also outlined in the JIS specification titled “Minimum Readable Text Size at Different Ages” for reference (see Figure 3).

When designing lighting for older adults' homes, reflected light should be used whenever possible. In addition, switches should have significant, visible indicators that are easy to locate in low light. Especially when the elderly go to the toilet at night, they often cannot locate the light switch in the darkness since the direct light is too harsh.

The majority of elderly people suffer from deafness, a condition that makes it necessary for them to speak louder in order to be clearly understood by others. This is the health problem that is most common among older people. The outer ear, the middle ear, and the inner ear are all components of the auditory system, which is a physiological process. The physiology of hearing is comprised of these three components in its entirety. Due to the natural process of aging, older people typically have a greater tendency to accumulate a significant amount of hard earwax in the external auditory canal. Both the hair cells of the cochlea and the cells that make up the auditory nerve pathway are susceptible to apoptosis and degeneration, which are both processes that can take place in these cell types. In addition, the blood supply to the cochlear cells of elderly people is typically insufficient. This can cause hearing loss. All of these factors play a role in hearing loss in older people, and the primary ways in which they manifest themselves are discussed in the paragraphs that follow.

The tone ought to have a lofty quality: hearing at 4 decibels and 6,000 Hz is possible for an adult who is 30 years old. A person who is 65 years old is required to raise the volume of the sound to a level of 40 decibels while maintaining the same frequency.

Decreased auditory selectivity: we are all familiar with the “cocktail party effect,” in which one person's conversation dominates the attention of the listener to the exclusion of all other conversations. As people get older, their ability to selectively process sound through their ears typically declines. Older people frequently have trouble hearing low notes and feel uneasy when exposed to high notes. They also tend to favor slower conversations over faster ones and prefer silence to noise.

Plan your actions to maximize the impact on the ear: it is possible for electronic products with voice alerts to avoid loud and piercing sounds while also maintaining sound frequencies that are within the hearing range of older people (see Table 2).

The natural process of aging has the effect of diminishing a person's capacity to recognize objects using their senses of touch, taste, and smell. This occurs as a result of the death of cells in the skin. As people get older, their skin cells degenerate, making it more difficult for them to feel both touch and pain. This is especially true for those who are elderly. People's sensory organ systems begin to degenerate as they get older, which results in a decline in a variety of sensory functions as people age. This includes a diminished capacity for touch and a diminished sense of smell. When a person reaches the age of sixty, their skin begins to show signs of aging such as wrinkles, age spots, atrophy of glands, and a reduction in the number of sweat glands. Additionally, the number of sensitive tactile points on the skin decreases during this time. The level of a perceptual stimulus that must be present in order for it to be interpreted by the brain as a cutaneous touch gradually increases as we get older. In addition, people as they age are more likely to suffer from injuries such as bruises and burns as a result of a diminished awareness of both temperature and pain.

In the year 1954, McGill University, which is located in Canada, was the site of a psychological experiment. Students were required to wear remarkable translucent plastic eyes (to simulate visual deprivation), cardboard gloves, and cuffs (to simulate tactile deprivation) and to maintain complete silence while in a specific room that was filled with repetitive humming sounds (auditory deprivation). After the experiment, the majority of the subjects reported feeling restless and reported that they did not last the full three days. They were unable to maintain their concentration, their logic became jumbled, they were unable to think normally, and as a result, their intelligence was significantly diminished. Deprivation of sensation will invariably have an effect on more complex and higher-level mental phenomena such as memory and reasoning, despite the fact that sensation is a relatively straightforward and low-level mental activity.

Because of this, the natural decline in physical health that comes with aging can also have an impact on a person's cognitive abilities.

The skeletal and muscular systems of elderly people experience a gradual deterioration that manifests itself as slower reactions, decreasing flexibility, decreased muscle strength, and decreased muscle control. Other signs of this deterioration include bone loss and joint stiffness. The peak of a person's muscular strength typically occurs between the ages of 20 and 30, after which it tends to decline, with a person's strength at age 70 being only half as muscular as it was at age 30. The peak of a person's cardiovascular strength typically occurs between the ages of 40 and 60, when it tends to remain relatively stable.

Walking, climbing stairs, and maintaining one's balance are all activities that require a certain amount of strength in the lower limbs. This strength is especially important for people who are getting older because these activities become more difficult with age. The findings of a number of studies indicate that around the age of 30, the body's muscle strength reaches its maximum level, after which it begins to gradually lose function. This phenomenon is known as “muscle atrophy.” A muscle will contract and change its organizational structure when the number of muscle fibers within it decreases. This will cause the muscle to shrink. The accumulation of additional body fat is the cause of the gradual loss of muscular strength, elasticity, tone, and speed that occurs during exercise. This loss is caused by the increased body fat.

The ability of a muscle group to contract at a maximum rate for an extended period of time is referred to as muscle endurance. On the other hand, the ability of a single muscle fiber to produce a contraction in response to an external force is referred to as muscle strength. Muscle endurance is greater than muscle strength. A significant decline in one's muscular strength and endurance can be the result of both advancing age and a lack of participation in physically active pursuits. According to William (1999), getting older is one of the most significant factors that can contribute to muscle atrophy. The natural process of getting older, when combined with a lack of physical activity, results in a gradual loss of muscle strength, which, in turn, results in decreased mobility and impaired movement. As a natural consequence of growing older, people in their later years are more likely to be hurt in incidents that are caused by accidents.

The natural process of aging is characterized by a gradual loss of muscle mass, which is the component that generates the most interest and debate. This condition is brought on by the interaction that takes place between the neurological and muscular systems as a result of a decrease in the amount of physical activity that a person gets. The number of muscle cells as well as the volume of those cells decreases with advancing age. The average age at which a person begins to experience a decline in their muscle mass is somewhere in the vicinity of the age of 50. Even though a decrease in muscle mass leads to a decrease in muscle strength, there is still a chance that moderate exercise can improve either muscle strength or muscle endurance. This is because a decrease in muscle mass causes a decrease in muscle mass. According to the findings of a study that was carried out by Tetsuo Fukunaga using ultrasound technology to measure the changes in muscle mass, there is a natural loss of three to five percent of muscle mass every ten years after the age of twenty-five. This loss of muscle mass occurs on a consistent basis. The strength of a person's knee extensors, knee flexors, dorsiflexion, plantar flexors, elbow extensors, and elbow flexors at the age of 70 was, respectively, 60%, 80%, 70%, 67%, 76%, and 87% of what it was when they were 20 years old. This information comes from some research.

## 4. Methods for Measuring Physical Quantities in Sensible Engineering

Table 3 shows that in today's world, modern life is accelerating, young people cannot always accompany the elderly due to the pressures of life, and consequently, the elderly will fall, lose, and become ill (see Figure 4). Therefore, artificial intelligence physiotherapy is essential for the elderly.

## 5. Analysis of Cognitive-Perceptual Imagery of the Elderly in Advanced Age

The term “cognitive functions” refers to the capabilities of an individual, or group of individuals, to recognize and reflect upon objective things. A person's attention, imagination, capacity for learning and memory, as well as their capacity for logical reasoning, are all examples of cognitive functions. The process of cognitive aging has the effect of making it more difficult for older people to take in new information, making it more difficult for older people to pay attention for longer periods of time, and making older people's memories less reliable as they get older. Memory loss can also cause a loss of the ability to perform activities of daily living, which can result in impaired logical reasoning, slower sensory analysis, and longer motor response times. Memory loss can also cause a loss of the ability to perform activities of daily living.

Attention is the capacity to concentrate on a specific stimulus despite the presence of other stimuli in the environment that vie for a share of our limited attentional resources. When we pay attention to a stimulus, we are able to acquire perception of that stimulus, whereas stimuli that are not the focus of our attention appear fuzzy and are misperceived as not being heard or seen.

Everyone has trouble concentrating at the moment because the Internet is fragmenting at this time, and as a result, they are forced to switch their attention due to the many different stimuli that come from the outside. When people get older, their bodies change in a way that makes them physiologically less attentive and less able to sustain attention. As a result, they lose the precision and speed that were necessary to exercise attention control when they were younger.

Language based on perceptual imagery: it can be difficult for older people to ignore information that is irrelevant or distracting if it is stored in their working memory because they have a tendency to have a short attention span that is both sticky and inert.

Memory is the mental phenomenon by which a person receives information and retains it afterward, and it is also the basis for learning a variety of human behaviors. Memory is the mental phenomenon by which a person receives information and retains it afterward. Memory serves as the foundation for the acquisition of a wide variety of human behaviors. Memory can be segmented into three distinct subtypes: short-term memory, long-term memory, and sensory memory. Sensory memory is defined as the ability to remember the effects of a sensory stimulus for an extended period of time after the stimulus has been removed. When watching a movie, the viewer's sensory memories enable them to perceive a still image that is being displayed at a rate of 24 frames per second as a continuous image. This occurs because the viewer's eyes and brain are working together to create this illusion. In the memory known as short-term memory, only bits and pieces of information are stored for a period of time that is no longer than a few seconds. For instance, the discipline of interaction design has a rule that is referred to as the “magic number 72 rule.” This rule states that people start making mistakes when they memorize 5-9 different chunks of information, and it has been around for quite some time. Something that is frequently brought to mind has the potential to be stored in the long-term memory, where it can be permanently retained and has a lower risk of being forgotten. When something is frequently brought to mind, it has the potential to be stored in the long-term memory (see Figure 5).

As we get older, we experience a decline in our short-term memory not because we are unable to effectively attend to or ignore information that is relevant, but rather because we are unable to effectively ignore information that is irrelevant, which leads to an overload of the limited capacity of our short-term memory.

Memory capacity begins to decline with increasing age, which is accompanied by a decline in numerical aspects and nonverbal dependent memory activities. Additionally, it takes a person longer to recall an event, and they store new memories less effectively than younger adults. In spite of this, senior citizens can still keep a strong memory of their memories by engaging in logical exercises like recalling the stories that their grandparents used to tell them when they were young.

Language based on perceptual imagery: to generate mental images, recitation and repetition are both essential components.

Thinking is the process of analyzing, comparing, synthesizing, generalizing, and abstracting, forming concepts, reasoning, and judgments based on the information obtained by sensory perception, and is the highest form of human cognitive activity.

With advancing age, the knowledge of the elderly diminishes, and in particular, the mind's ability to be agile, fluent, flexible, unique, and creative is less than it was in youth.

Sensual imagery language: the aging process causes deterioration in perception and memory, accompanied by loss of concepts, logical reasoning, and problem-solving skills.

Following is an analysis of cognitive-perceptual imagery of elderly people who have reached advanced age. This analysis identifies the primary factors that determine the imagery of interactive design. Because of this, designers will be able to formulate a strategy for the interactive design of the future. Using multiple regression analysis, a correlation between somatosensory and perceptual elements as well as perceptual evaluation was investigated, and the relationship between the three was summarized.  Figure 6 provides a visual representation of the Kansei Engineering System (KES) research methodology. Different products will emerge that are a reflection of the thoughts of users as a result of the analysis of perceptual factors, and the development of new technologies will be based on the physiological and psychological factors of human beings. You can put your faith in the fact that senior citizens will be given more consideration in the twenty-first century.

The artificial intelligence physiotherapy robot that is standardized has access to an exceptional pool of expertise, cutting-edge scientific testing, monitoring equipment, and conditioning tools. “Precision physiotherapy” can be accomplished by robots with artificial intelligence, leading to significant improvements in the physical condition of less healthy populations. When compared to the benefits of manual physiotherapy, the advantages of artificial intelligence physiotherapy are in a league of their own. They will almost certainly result in significant shifts in the way that the environment public health physiotherapy industry delivers its services, which is of utmost importance for ensuring the continued growth of the environment public health industry's commitment to providing services of the highest possible standard.

## 6. Conclusion

According to the findings of the research and analysis that were presented earlier, the cis-perceptual engineering system, also known as sensual physical data, is an efficient tool for designers who are creating sensual products, as demonstrated in Figure 7.

The economic status of the target demographic, the spending power of that demographic, the aesthetic preferences of that demographic, the behavioral patterns of that demographic, the product brand awareness of that demographic, market trends, and any other essential background information for the design make up the macroproduct factors. Analysis of the semantics of macroscopic product perceptions can be accomplished through the use of cis-perceptual engineering.

The macroproduct factors include the target group's economic status, spending power, aesthetic preferences, behavioral habits, product brand awareness, market trends, and other essential background information for the design. Cis-perceptual engineering is used to analyze the semantics of macroscopic product perceptions.

## Figures and Tables

**Figure 1:** Scope of artificial intelligence, machine learning, and deep learning.

**Figure 2:** Three stages of artificial intelligence development.

**Figure 3:** Minimum readable text size for different ages.

**Figure 4:** The Elderly and Their Aging, Demographic Sourcebook, Institute of Population Studies, Ministry of Health and Welfare, Japan.

**Figure 5:** Memory schematic.

**Figure 6:** Perceptual analysis of the image of the aged.

**Figure 7:** Schematic diagram of hybrid inductive engineering.

**Table 1:** Diseases of the elderly due to the degree of blurred vision.

The elderly cause of blurred vision		
Pathogeny	Low vision	Blind
Presbyopia	√	
Senile cataract	√	√
High myopia	√	√
Age related macular degeneration	√	√
Diabetes retinopathy	√	
Glaucoma	√	
Keratopathy	√	
Atrophy of eyeball and optic nerve	√	√

**Table 2:** Comparison of pure tone hearing threshold and speech intelligibility in the elderly with the young (dB HL, *x* ± *s*).

Group	Number of ears	PTA	4.8 kHz	4 kHz	PB max
			Average hearing threshold	Average hearing threshold	(%)
Young group 1	30	6.67 ± 4.82	7.08 ± 5.49	7.33 ± 5.28	95.60 ± 3.20
Elderly group A					
I	15	14.28 ± 5.70	22.80 ± 5.4	19.69 ± 5.40	92.80 ± 4.10
II	29	17, 66 ± 3.51	45.17 ± 6.95	38.83 ± 9.55	92.67 ± 4.21
III	9	19.99 ± 2.22	74.17 ± 10.80	74.44 ± 11.19	83.56 ± 7.66
IV	17	30.99 ± 3.87	51.6 ± 7.03	49.33 ± 7.72	87.53 ± 6.93
V	13	29.75 ± 5.38	71.73 ± 5.98	66.92 ± 8.67	85.00 ± 9.4
VI	8	46.29 ± 3.50	70.83 ± 7.34	70.63 ± 10.73	70.25 ± 13.10
VII	9	61.84 ± 8.09	84.58 ± 6.73	80.00 ± 10.54	62.30 ± 6.50

**Table 3:** Physical and mental functional status of the elderly, the concept of residential planning for the elderly, Chen Zhengxiong, 2004.

Aging condition	Primary aging	Secondary aging	Tertiary aging
Physical and mental condition	Health period	Obstacle period	Ambulatory period
Degree of movement	Can run, jump, walk	Need assistive devices such as crutches and wheelchairs	Almost bedridden
Distribution ratio (%)	75%	20%	5%
Living ability	Have self-care ability	Need to be taken care of by others	

## Data Availability

The dataset used to support the findings of this study are available from the corresponding author upon request.

## References

[1] Qian K., Zhang Z., Yamamoto Y., Schuller B. W. (2021). Artificial intelligence internet of things for the elderly: from assisted living to health-care monitoring. *IEEE Signal Processing Magazine*.

[2] Nahian M., Ghosh T., Uddin M. N., Islam M., Mahmud M., Kaiser M. S. (2020). Towards Artificial Intelligence Driven Emotion Aware Fall Monitoring Framework Suitable for Elderly People with Neurological Disorder. *International Conference on Brain Informatics*.

[3] Méndez J. I., Mata O., Ponce P., Meier A., Peffer T., Molina A. (2020). Multi-Sensor System, Gamification, and Artificial Intelligence for Benefit Elderly People. *Challenges and Trends in Multimodal Fall Detection for Healthcare*.

[4] Vercelli A., Rainero I., Ciferri L., Boido M., Pirri F. (2018). Robots in elderly care. *Digit Cult-Scientific Journal on Digital Cultures*.

[5] Porkodi S., Kesavaraja D., Dubey A. K., Kumar A., Kumar S. R., Gayathri N., Das P. (2021). Healthcare robots enabled with IoT and artificial intelligence for elderly patients. *In AI and IoT-Based Intelligent Automation in Robotics*.

[6] Rong J., Ji X., Fang X., Jee M. H. (2022). Research on material design of medical products for elderly families based on artificial intelligence. *Applied Bionics and Biomechanics*.

[7] Xiong J., Ma T., Lian Z., de Dear R. (2019). Perceptual and physiological responses of elderly subjects to moderate temperatures. *Building and Environment*.

[8] Kemp B. J. (1973). Reaction time of young and elderly subjects in relation to perceptual deprivation and signal-on versus signal-off conditions. *Developmental Psychology*.

[9] Waldock K. A. M., Hayes M., Watt P. W., Maxwell N. S. (2018). Physiological and perceptual responses in the elderly to simulated daily living activities in UK summer climatic conditions. *Public Health*.

[10] de Menezes K. S., Master S., Guzman M., Bortnem C., Ramos L. R. (2014). Diferencias de los parametros acusticos y perceptuales de la voz entre sujetos ancianos y jovenes con intensidad habitual y alta. *Acta Otorrinolaringologica*.

[11] Botchweynisha D., Trowbridgematthew F. (2014). Green health. *Journal of Planning Education and Research*.

[12] Shi W. X., Liu M. C. (2012). Telemedicine information demands of Chinese elderly people in the future: examination of effectiveness in applications. *Applied Mechanics and Materials*.

[13] Kim S.-G., Lee J.-H. (2019). The artificial intelligence based usability testing techniques for elderly person. *Basic & clinical pharmacology & toxicology*.

[14] Al Nahian M. J., Ghosh T., Uddin M. N., Islam M. M., Mahmud M., Kaiser M. S. (2020). Towards Artificial Intelligence Driven Emotion Aware Fall Monitoring Framework Suitable for Elderly People with Neurological Disorder. *Brain informatics: 13th international conference on brain informatics (BI)*.

[15] Saarela M., Ryynanen O.-P., Ayramo S. A. M. I. (2019). Predicting hospital associated disability from imbalanced data using supervised learning. *Artificial Intelligence in Medicine*.

[16] Gandhi S., Goyal A. (2021). The Jet-I-U: a biomimetic assistive robot for the visually impaired and elderly. *International journal of hybrid intelligent systems*.

[17] Ravi D., Wong C., Deligianni F. (2017). Deep learning for health informatics. *IEEE Journal of Biomedical and Health Informatics*.

[18] Noorbakhsh-Sabet N., Zand R., Zhang Y., Abedi V. (2019). Artificial intelligence transforms the future of health care. *The American Journal of Medicine*.

[19] Caic M., Odekerken-Schroder G., Mahr D. (2018). Service robots: value co-creation and co-destruction in elderly care networks. *Journal of service management: JOSM*.

[20] Davies N. (2016). Can robots handle your healthcare?. *Engineering & technology: E & T: IET engineering & technology*.

